The article "Nuclear factor of activated T cells 5 maintained by Hotair suppression of miR-568 upregulates S100 calcium binding protein A4 to promote breast cancer metastasis" was retracted in 2018. Reason: duplicated images.

# Nuclear factor of activated T cells 5 maintained by Hotair suppression of miR-568 upregulates S100 calcium binding protein A4 to promote breast cancer metastasis

**DOI:** 10.1186/s13058-014-0454-2

**Published:** 2014-10-14

**Authors:** Jun-Tang Li, Li-Feng Wang, Ya-Li Zhao, Tao Yang, Wei Li, Jing Zhao, Feng Yu, Lei Wang, Yan-Ling Meng, Ning-Ning Liu, Xiao-Shan Zhu, Chun-Fang Gao, Lin-Tao Jia, An-Gang Yang

**Affiliations:** 1 State Key Laboratory of Cancer Biology, Department of Immunology, Fourth Military Medical University, Xi’an, 710032 Shaanxi China; 2 Institute of Anal-Colorectal Surgery, No. 150 Central Hospital of PLA, Luoyang, 471000 Henan China; 3 Department of Biochemistry and Molecular Biology, Fourth Military Medical University, Xi’an, 710032 Shaanxi China

## Abstract

**Introduction:**

The onset of distal metastasis, which underlies the high mortality of breast cancers, warrants substantial studies to depict its molecular basis. Nuclear factor of activated T cells 5 (NFAT5) is upregulated in various malignancies and is critically involved in migration and invasion of neoplastic cells. Nevertheless, the metastasis-related events potentiated by this transcriptional factor and the mechanism responsible for NFAT5 elevation in carcinoma cells remain to be fully elucidated.

**Methods:**

The correlation of NFAT5 with breast cancer invasiveness was investigated *in vitro* and clinically. The genes transcriptionally activated by NFAT5 were probed and their roles in breast cancer progression were dissected. The upstream regulators of NFAT5 were studied with particular attempt to explore the involvement of non-coding RNAs, and the mechanism underlying the maintenance of NFAT5 expression was deciphered.

**Results:**

In metastatic breast cancers, NFAT5 promotes epithelial-mesenchymal transition (EMT) and invasion of cells by switching on the expression of the calcium binding protein S100A4, and facilitates the angiogenesis of breast epithelial cells and thus the development of metastases by transcriptionally activating vascular endothelial growth factor C (VEGF-C). NFAT5 is directly targeted by miR-568, which is in turn suppressed by the long non-coding RNA, Hotair, via a documented *in trans* gene silencing pattern, that is recruitment of the polycomb complex (Polycomb Repressive Complex 2; PRC2) and LSD1, and consequently methylation of histone H3K27 and demethylation of H3K4 on the miR-568 loci.

**Conclusion:**

This study unravels a detailed role of NFAT5 in mediating metastatic signaling, and provides broad insights into the involvement of Hotair, in particular, by transcriptionally regulating the expression of microRNA(s), in the metastasis of breast cancers.

The article "Nuclear factor of activated T cells 5 maintained by Hotair suppression of miR-568 upregulates S100 calcium binding protein A4 to promote breast cancer metastasis" was retracted in 2018. Reason: duplicated images.

**Electronic supplementary material:**

The online version of this article (doi:10.1186/s13058-014-0454-2) contains supplementary material, which is available to authorized users.

## Introduction

Distal metastasis is the leading cause of mortality in breast cancer patients [1]. The migration of neoplastic cells from primary tumors to target organs occurs through a complex series of steps driven by divergent molecules that interact to control cell motility and invasiveness [2],[3]. Briefly, metastatic cells detach from the tumor mass, intravasate into the blood or lymph vessels, extravasate into surrounding tissues, and colonize appropriate organ sites [2]-[4]. Numerous cytoskeleton-interacting proteins, adhesion molecules, chemotactic factors, and extracellular matrix proteins such as the matrix metalloproteinases (MMPs) are involved in the invasion of cancer cells, representing a common molecular machinery of metastasis [5],[6]. However, the upstream driver signals culminating in activation of this machinery remains largely uncharacterized [5],[6].

Diverse transcription factor families, including the nuclear factors of activated T cells (NFATs), have been shown to play essential roles in regulating the expression of metastasis-related proteins [7]-[9]. Accumulating evidence suggests that NFAT5, which was originally identified for its involvement in osmotic cellular stress and adaptation, plays a pivotal role in cancer cell migration [8],[10]. Nevertheless, the mechanism by which NFAT5 mediates metastasis is not fully deciphered, nor are the signals that dictate NFAT5 expression in metastatic breast cancers. Here, we show that in metastatic breast cancers, NFAT5 is abundantly expressed, and the upregulated NFAT5 transcriptionally activates the calcium-binding protein S100A4 and vascular endothelial growth factor C (VEGF-C). Given the well-established role of S100A4 in regulating the expression of so-called metastasis executioners like MMPs, as well as the critical involvement of VEGF-C in regulating cell adhesion, permeability of blood and lymph vessels, and angiogenesis of tumors, NFAT5 is likely involved as a key player in promoting the invasion of breast cancer cells and formation of distal metastases [11],[12].

The imperative regulatory role of non-coding RNAs in the development and progression of cancer has been documented [13]. Of note are microRNAs (miRNAs), which posttranscriptionally inhibit target genes, and long non-coding RNAs (lncRNAs) such as Hotair, which is critically involved in cancer metastasis by extensively remodeling the chromosomal loci of multiple metastasis-related genes [14],[15]. In addition to *in cis* control of the HOX family genes, Hotair modulates the expression of a variety of genes *in trans* by recruiting components of the polycomb complex PRC2 and the LSD1/CoREST/REST complex, thus orchestrating histone H3K27 trimethylation and H3K4 demethylation and consequently triggering epigenetic gene silencing [13]. While candidate Hotair-responsive genes have been identified by a systemic investigation based on Hotair-induced PRC2 and LSD1 occupancy, it is unclear whether miRNAs act in concert with the lncRNAs or as targets of the lncRNAs in mediating metastasis-related signaling [14],[16],[17]. We found in metastatic breast cancers that NFAT5 is a direct target of miR-568, which is in turn suppressed by Hotair via PRC2 recruitment and subsequent chromosomal silencing of the miR-568 gene. Thus, NFAT5 is among the candidate mediators of Hotair-driven transcriptional activation of metastasis-related genes in breast cancer.

The article "Nuclear factor of activated T cells 5 maintained by Hotair suppression of miR-568 upregulates S100 calcium binding protein A4 to promote breast cancer metastasis" was retracted in 2018. Reason: duplicated images.

## Methods

### Culture and transfection of breast cancer cell lines

The human breast cancer cell lines MDA-MB-231, MDA-MB-453, MDA-MB-468, BT549, MCF-7, T47D, SKBr-3, and Bcap37 were purchased from the Cell Bank of Shanghai Institute for Biological Sciences, Chinese Academy of Sciences. All cell lines were characterized by gene profiling analysis by the provider, and were used fewer than 6 months after receipt. Cells were cultured in Dulbecco’s modified Eagle’s medium (DMEM) containing 10% FBS, and maintained at 37°C in a humidified atmosphere containing 5% CO_2_. The miR-568 mimic, antagomiR-568, and siRNAs were synthesized by GenePharma (Shanghai, China). Transfection of cells was performed using Lipofectamine 2000 reagent (Invitrogen/Life Technologies, Carlsbad, CA, USA), according to the manufacturer’s instructions.

### Lentiviral expression of miRNA or shRNA

Short hairpin RNAs (shRNAs) were designed to target NFAT5 using scrambled shRNA as a control. Paired deoxyribonucleotide oligos encoding the shRNAs were synthesized, annealed, and cloned into the *Eco*RI and *Nco*I sites of the pLKO.1 vector (Addgene, Cambridge, MA, USA). The above constructs were co-transfected into HEK293T cells with the lentivirus packaging plasmids pCMV-VSVG and pCMV-ΔA.9. The virus in conditioned medium was harvested, filtered, and used for infection of breast cancer cells. Cells were selected with puromycin (5 μg/mL) for the generation of stable shRNA-expressing clones. For lentiviral expression of miR-568, complementary DNA strands corresponding to the pre-miR-568 sequence were synthesized and cloned into the AgeI and EcoRI sites of pGCsi-H1-CMV-GFP (GeneChem, Shanghai, China). The recombinant or empty vector was co-transfected with the packaging plasmids pMD2.G and psPAX2 into HEK293T cells. The virus-containing medium was harvested, filtered, and used for infection.

The article "Nuclear factor of activated T cells 5 maintained by Hotair suppression of miR-568 upregulates S100 calcium binding protein A4 to promote breast cancer metastasis" was retracted in 2018. Reason: duplicated images.

### Quantitative reverse transcription (RT)-PCR

Total RNA was extracted from cells using TRIzol reagent (Invitrogen/Life Technologies) according to the manufacturer’s protocol. Reverse transcription was performed using SuperScriptTM II Reverse Transcriptase (Invitrogen/Life Technologies), and cDNAs were amplified and detected using SYBR Premix Ex TaqTM (TaKaRa, Otsu, Shiga, Japan). To quantify miRNAs, total RNA was reverse-transcribed using the miScript Reverse Transcription Kit (Qiagen, Hilden, Germany) and then amplified using SYBR Premix Ex TaqTM (TaKaRa). Primers used for PCR amplification are provided in Additional file 1: Table S1.

### Western blotting

Cells were harvested at the desired times, and proteins were extracted, separated on an SDS/PAGE gel, transferred onto polyvinylidene fluoride membranes, and subjected to immunoblot analyses. Blotting was performed using antibodies targeting NFAT5 (Abcam, Cambridge, UK), S100A4, E-cadherin, vimentin (all from Abnova, Taiwan, China), α-catenin (Santa Cruz, Dallas, TX, USA), β-catenin, Akt, phosphorylated Akt, ERK, phosphorylated ERK (all from Cell Signaling Technology, Danvers, MA, USA), and β-actin (Sigma-Aldrich, St. Louis, MO, USA).

### ELISA assay

VEGF-C protein in culture medium or patient peripheral blood samples was measured using a human VEGF-C ELISA kit (Boster, Wuhan, China). VEGF-C concentration expressed as pg/mL was calibrated against a highly purified recombinant human VEGF-C. Briefly, 1 mL of medium was centrifuged at 12,000 r/minute for 5 minutes at 4°C, and 200 μL of supernatant was used in the ELISA according to the manufacturer’s instructions. The optical absorbance of the samples was measured at 490 nm using a microplate reader (Bio-Rad). A serial dilution of human recombinant VEGF-C was included in each assay to obtain a standard curve from which the sample values of VEGF-C were extrapolated.

### Luciferase reporter assay

The 3′UTR of wild-type NFAT5 and a variant containing mutations in the putative miR-568 binding sites were inserted downstream of the firefly luciferase gene in the pGL3 vector (Promega, Madison, WI, USA). HEK293 cells were co-transfected with reporter constructs, an internal control vector (pGL4.73), and a synthetic miR-568 mimic. At 48 h after transfection, luciferase activity was assayed using the Dual-Luciferase Reporter Assay System (Promega) and a luminometer (Glomax 20/20, Promega), and normalized to the activity of Renilla luciferase driven by a constitutively expressed promoter in the phRL vector. Basal promoter activity was measured as the fold-change relative to the activity observed with the basic pGL3 vector alone.

The article "Nuclear factor of activated T cells 5 maintained by Hotair suppression of miR-568 upregulates S100 calcium binding protein A4 to promote breast cancer metastasis" was retracted in 2018. Reason: duplicated images.

### Chromatin immunoprecipitation

MDA-MB-231 cells were crosslinked with formaldehyde and harvested for chromatin immunoprecipitation (ChIP) as described [18]. Briefly, chromatin was fragmented by sonication, and pre-cleared chromatin was immunoprecipitated overnight with monoclonal antibodies against NFAT5 (Abcam, UK), EZH2 (Millipore, Darmstadt, Germany), LSD1 (Abcam), trimethylated histone H3K27 (Millipore), dimethylated histone H3K4 (Abnova) or corresponding IgG isotype control (Abcam). The enrichment of specific DNA fragments was analyzed by PCR with primers flanking the S100A4, VEGF-C or miR-568 promoter region.

### Immunofluorescence and immunohistochemistry

MDA-MB-231 cells were grown on glass coverslips and were allowed to attach for 24 h prior to staining. The coverslips were washed, fixed in 3.7% (wt/vol) formaldehyde, immersed sequentially in cold methanol and cold acetone, and then allowed to air dry. The dry coverslips were incubated with diluted antibodies against E-cadherin or vimentin (Abnova), followed by incubation with a Cy3- or fluorescein isothiocyanate-conjugated secondary antibody. The nuclei were counter-stained with 4′,6-diamidino-2-phenylindole (DAPI). The coverslips were mounted with Aqua-mount (Lerner Laboratories, USA) for immunofluorescent microscopy.

The strepavidin-peroxidase (SP) method was used to detect the expression of genes of interest in clinical breast cancer samples by immunohistochemistry. Briefly, tissues were sectioned, treated with 3% H_2_O_2_, and then incubated in 5% goat antiserum. Primary antibodies against NFAT5 (Abcam), S100A4 (Abnova), E-cadherin (Abnova) or vimentin (Abnova) were added to serial tissue sections and incubated overnight, followed by incubation with a biotin-labeled secondary antibody. SP complex was added and then DAB-H_2_O_2_ was used for the color reaction before microscopy.

### *In vitro*cell migration and invasion assays

For the cell motility assay, trypsinized cells were resuspended in serum-free RPMI 1640 medium supplemented with 0.1% bovine serum albumin (BSA). Cell suspensions were seeded in the upper chamber of a transwell insert with an 8 μm diameter (Corning, Tewksbury, MA, USA), and complete medium was added to the lower chamber. After incubation for 24 h, cells on top of the membrane were displaced with a cotton swab, and cells on the bottom of the membrane were fixed in methanol and stained with crystal violet. Cells in three fields were counted per membrane. For the invasion assay, the transwell was coated with 200 μL Matrigel at 200 μg/mL and pre-incubated with RPMI1640 medium. Cells were seeded into the upper chamber of the transwell (20,000 cells/insert) and RPMI 1640/BSA was added to the lower chamber. After 24 h of incubation at 37°C, cells were fixed in methanol and stained with crystal violet or DAPI. Cells that invaded through the pores to the lower surface of the filter were counted under a microscope. Three invasion chambers were used per condition, and the total number of cells from the three filters was averaged. For the wound-healing assay, 1 × 10^6^ cells were seeded on 6-cm plates coated with 10 μg/mL type I collagen. Cells were incubated for 24 h, the monolayer was disrupted with a cell scraper (1.2 mm width), and photographs were taken at 0 and 24 h with a phase-contrast microscope. Experiments were carried out in triplicate, and four fields of each condition were recorded.

The article "Nuclear factor of activated T cells 5 maintained by Hotair suppression of miR-568 upregulates S100 calcium binding protein A4 to promote breast cancer metastasis" was retracted in 2018. Reason: duplicated images.

### *In vitro*tube formation assay

Human umbilical vein endothelial cells (HUVECs) were obtained from the Institute of Biochemistry and Cell Biology, Chinese Academy of Sciences. Cells were co-cultured with breast cancer cells using a double-chamber method in 24-well plates as described [19]. MDA-MB-231 cells (1 × 10^4^ cells) were seeded into transwell chambers consisting of polycarbonate membranes with 0.45-μm pores and allowed to adhere overnight. The chambers were then placed into the HUVEC culture and were co-cultured for 4 to 8 days. Medium of HUVECs was removed and the collagen gel prepared as previously described [19] was applied to the cells. Fresh DMEM containing 3% FBS was then added to the collagen gel and cells were incubated at 37°C for 24 h. The reorganization of the subconfluent monolayer HUVECs was monitored and photographed with a phase contrast microscope (Nikon).

### *In vivo*tumor growth and metastasis assay

Female, 5- to 7-week-old BALB/c nude mice (Institute of Zoology, Chinese Academy of Sciences) were injected subcutaneously into the right hind flank with 10^6^ MDA-MB-231 cells infected with control lentivirus or recombinant lentivirus expressing an NFAT5-targeting or a scrambled shRNA (n =5 mice/group). Tumor volume was monitored and calculated as follows:

$$\mathrm{Tumor}\;\mathrm{volume}\;=\;\mathrm{Widt}h^{2}\;\times \;\mathrm{Length}/2\text{.}$$

All mice were sacrificed at 7 weeks post-inoculation, and tumors were removed and weighed.

For the metastasis assays, MDA-MB-231 cells infected with control lentivirus or recombinant lentivirus expressing an NFAT5-targeting shRNA, a scrambled shRNA, or a miR-568 precursor were used for *in vivo* metastasis assays (n =5 mice/group). Female 5- to 7-week-old BALB/c nude mice were injected through the tail vein with 10^6^ cells. The mice were monitored for general health status and evidence of morbidity related to the primary tumor or metastasis. Mice were sacrificed at 7 weeks post inoculation, and anatomized mice were examined for metastasis in the lung or lymph nodes. Lungs and other organs with visible tumor colonies were fixed and embedded in paraffin, and three non-sequential serial sections per animal were obtained. The sections were stained with hematoxylin/eosin and analyzed for the presence of metastasis by light microscopy. The total number of metastases per lung section was counted and averaged. All of the above animal experiments were approved by the Committee of Laboratory Animal Care of the Fourth Military Medical University.

The article "Nuclear factor of activated T cells 5 maintained by Hotair suppression of miR-568 upregulates S100 calcium binding protein A4 to promote breast cancer metastasis" was retracted in 2018. Reason: duplicated images.

### Clinical sample collection

Breast cancer, normal breast tissue and venous blood samples were collected from Xijing Hospital, Fourth Military Medical University, China. Briefly, breast cancer samples from 30 patients were collected immediately after surgical resection in the Department of Vascular and Endocrine Surgery. All patients received surgery in 2010 without prior chemotherapy or radiotherapy. All cases were confirmed by hematoxylin/eosin staining, and pathological analysis revealed 8 patients with invasive lobular carcinoma and 22 with invasive ductal carcinoma. The diameter of the primary tumor was ≤2 cm in 11 patients and >2 cm in 19 patients. According to the tumor, node, metastasis (TNM) classification system of the Union for International Cancer Control (UICC), 21 and 9 cases were at stages I/II and III/IV, respectively. Four normal breast tissue samples were obtained from patients undergoing breast reduction surgery in the Institute of Plastic Surgery, Xijing Hospital. The samples were then subjected to qRT-PCR or immunohistochemical analysis as described above. Patient survival time was calculated from the date of breast cancer diagnosis to the date of death or the last follow up.

Venous blood samples from 10 healthy volunteers, 20 patients with benign breast lesions, and 36 breast cancer patients were collected from the Department of Oncology, Xijing Hospital. No patients received chemotherapy, radiation, or hormone therapy. Twelve of the breast cancer patients were diagnosed with lymph node metastasis. The concentration of VEGF-C was measured by ELISA as described above.

All sample collections were obtained with consent from patients for participation in the study and publication of the results, and were approved by the Ethics Committee of the Fourth Military Medical University.

### Statistical analysis

Statistical analyses were performed using SPSS version 16.0 (SPSS Inc., Chicago, USA) for Windows. Student’s *t*-test was used to analyze results expressed as the mean ± SD, the Chi-squared test was used for the evaluation of frequencies, and the Kruskal-Wallis test was used for comparisons of more than two independent groups. The Pearson correlation test was used to determine the strength of the relationships between Hotair and miR-568 expression in clinical samples. Differences were considered significant when the *P*-value was less than 0.05.

The article "Nuclear factor of activated T cells 5 maintained by Hotair suppression of miR-568 upregulates S100 calcium binding protein A4 to promote breast cancer metastasis" was retracted in 2018. Reason: duplicated images.

## Results

### NFATcorrelates with high invasiveness of breast cancer cells

Given the documented involvement of NFATs in carcinogenesis and metastasis, we first analyzed in breast cancers the expression of NFAT5, a newly defined but evolutionarily oldest member of the family [7]-[9]. As a result, abundant NFAT5 was detected exclusively in breast cancer cell lines with high invasive potential (Figure 1A). In an attempt to determine the role of NFAT5 in the invasion of breast cancer cells, we silenced NFAT5 using small interfering RNAs (siRNAs) (Figure 1B). We found that knockdown of NFAT5 in highly metastatic breast carcinoma MDA-MB-231 cells significantly suppressed cell invasion and migration in transwell and wound-healing assays (Figure 1C and D). MDA-MB-231 cells modified to express NFAT5-targeting short hairpin RNA (shRNA) were next generated. While the formation and growth of primary xenograft tumors were comparable (data not shown), tumors developed from these cells showed significantly lower potential of lung metastasis in a xenograft model than that of tumors derived from control MDA-MB-231 cells (Figure 1E). In addition, NFAT5 exhibited significantly high expression in clinical breast carcinoma samples with detected metastases when compared with non-metastatic malignancies or normal breast tissues (Figure 1F). Thus, NFAT5 is involved in regulating the invasiveness of breast cancer cells.

**Figure 1:** **Nuclear factors of activated T cells 5 (NFAT5) dictates the invasiveness of breast cancer cells. (A)** qRT-PCR (upper panel) and western blotting (lower panel) assays for NFAT5 expression in breast cancer cell lines. Relative levels compared with the normal human mammary epithelial MCF-10A cells were plotted for qRT-PCR. **(B)** qRT-PCR and western blotting assays of MDA-MB-231 cells after transfection with control (100 nM) or NFAT5-targeted siRNAs. siNFAT5-2 was used thereafter due to its high efficacy in posttranscriptionally suppressing NFAT5 expression. **(C**, **D)** Transwell **(C)** and wound-healing **(D)** assays of cells transfected with scrambled or NFAT5-targeting siRNA. **(E)** MDA-MB-231 cells were modified with lentiviruses expressing scrambled or NFAT5-targeting shRNAs, and were injected into the tail vein of nude mice (n =10). The formation of lung metastases were monitored and representative H&E-stained lung tissues are shown. **(F)** qRT-PCR assay of 30 breast cancer samples (13 with metastases) and normal mammary tissues from four women undergoing breast reduction surgery. NFAT5 levels normalized to glyceraldehyde-3-phosphate dehydrogenase (GAPDH) are plotted. All data are representative photographs or represent the mean ± SD of three replicates. *P <0.05, **P <0.01. VEGF-C: vascular endothelial growth factor C.

The article "Nuclear factor of activated T cells 5 maintained by Hotair suppression of miR-568 upregulates S100 calcium binding protein A4 to promote breast cancer metastasis" was retracted in 2018. Reason: duplicated images.

### NFAT5 transcriptionally activates S100A4 and VEGF-C

NFAT5 has been reported to transcriptionally activate the cell motility and invasion regulator S100A4/metastasin, which is involved in integrin α6β4 signaling [7],[20]. Meanwhile, as a transcription factor initially identified for its vital role in osmotic stress, NFAT5 may regulate the expression of a cohort of genes that control vascular permeability [8],[21]. Consistent with these reports, S100A4 and VEGF-C showed similar expression patterns to NFAT5 in breast cancer cell lines with varied invasiveness (Figure 2A and B, Figure 1A and B). In accordance with cellular levels of NFAT5, abundant expression of S100A4 and VEGF-C were detected in highly metastatic MDA-MB-231 cells but not MCF-7 cells which is a non-invasive cell line (Figure 2C). Knockdown of NFAT5 resulted in substantial decrease in the cellular level of S100A4 as well as the expression and secretion of VEGF-C (Figure 2D and E). The binding of NFAT5 to the regulatory regions of the S100A4 and VEGF-C loci was confirmed by chromatin immunoprecipitation (ChIP) using an NFAT5 antibody (Figure 2F). Thus, S100A4 and VEGF-C are transcriptionally activated by NFAT5 in metastatic breast cancer cells.

**Figure 2:** **S100A4 and vascular endothelial growth factor C (VEGF-C) are transcriptionally activated by nuclear factors of activated T cells 5 (NFAT5). (A)** qRT-PCR assays of the indicated transcripts in breast cancer cell lines. Relative levels compared with MCF-10A cells were plotted. **(B)** Western blotting analysis (left) and ELISA quantification (right) of cellular S100A4 and secreted VEGF-C, respectively, in the indicated cell lines. **(C)** RT-PCR (left), western blotting (S100A4) and ELISA (secreted VEGF-C) assays for indicated gene expression. **(D**, **E)** RT-PCR **(D)**, western blotting and ELISA **(E)** assays for gene expression and after transfection of MDA-MB-231 cells with indicated siRNAs. **(F)** Chromatin immunoprecipitation (ChIP) assay using the lysates of indicated breast cancer cells. All data are representative photographs or represent the mean ± SD of three replicates. *P <0.05.

### NFAT5/S100A4 promotes invasion of breast cancer cells via epithelial-mesenchymal transition (EMT)

The involvement of S100A4 in NFAT5-mediated invasion of breast cancer cells was next evaluated. Comparable to NFAT5 silencing, knockdown of S100A4 impaired the invasion of cultured breast cancer cells (Figure 3A). The aforementioned executioners of metastasis involved in cell adhesion, migration and matrix degradation, in particular, CD44, RhoA, MMP2 and MMP9 were downregulated by siRNAs targeted to NFAT5 or S100A4 (Figure 3B). EMT is a hallmark of metastatic neoplasms, including breast cancers [22]. As expected, knockdown of S100A4 enhanced mutual adhesion of cultured MDA-MB-231 cells and induced a transition toward an epithelium-like morphology (Figure 3C). Concurrent upregulation of epithelial makers, such as E-cadherin and α-catenin, and downregulation of mesenchymal markers, such as vimentin, β-catenin, and Bmi1 were observed in breast cancer cells upon ablation of NFAT5 or S100A4 (Figure 3D to F). In advanced clinical breast cancer samples, high NFAT5 and S100A4 expression correlated with decreased E-cadherin but elevated vimentin levels (Figure 3G). These results suggest indispensable roles for S100A4 and EMT in NFAT5-mediated metastasis of breast cancers.

The article "Nuclear factor of activated T cells 5 maintained by Hotair suppression of miR-568 upregulates S100 calcium binding protein A4 to promote breast cancer metastasis" was retracted in 2018. Reason: duplicated images.

**Figure 3:** **Nuclear factors of activated T cells 5 (NFAT5)/S100A4 expedites epithelial-mesenchymal transition (EMT) and invasion of breast cancer cells. (A)** Transwell assay for the invasiveness of cells transfected with siRNAs targeting the indicated genes. **(B)** qRT-PCR assays for the expression of metastasis-related genes in MDA-MB-231 cells transfected with indicated siRNAs. Relative mRNA levels compared with untransfected cells were plotted. NC, scrambled negative control of siS100A4. **(C)** Microscopy of MDA-MB-231 cells showing suppressed spreading and increased intercellular contact upon introduction of S100A4-targeting siRNA. **(D** to **F)** Fluorescent microscopy **(D)**, western blotting **(E)** and qRT-PCR **(F)** assays of MDA-MB-231 cells after transfection with siRNAs targeting the indicated genes. **(G)** Representative photographs of immunohistochemical staining of breast cancers in clinical stages I to IV. Relative levels compared with untransfected cells were plotted for qRT-PCR assays in **(B)** and **(F)**. All data are representative images or represent the mean ± SD of three replicates. *P <0.05.

### NFAT5/VEGF-C signaling is involved in breast cancer metastasis

The formation and enlargement of metastatic foci, which usually dictate the prognosis of breast cancers, may rely on effective angiogenesis, prompting a potential role of sustained VEGF-C production in distal metastasis [12]. Indeed, we found that knockdown of NFAT5 or VEGF-C in MDA-MB-231 cells disrupted the formation of capillary-like tubes by co-cultured epithelial cells (Figure 4A). In clinical breast cancer samples, the expression of VEGF-C was significantly associated with breast cancer development and advanced-stage disease, and correlated well with the incidence of metastasis (Figure 4B to D). These results suggest that VEGF-C downstream of NFAT5 plays an essential role in breast cancer metastasis.

The article "Nuclear factor of activated T cells 5 maintained by Hotair suppression of miR-568 upregulates S100 calcium binding protein A4 to promote breast cancer metastasis" was retracted in 2018. Reason: duplicated images.

**Figure 4:** **Vascular endothelial growth factor C (VEGF-C) is involved in nuclear factors of activated T cells 5 (NFAT5)-driven progression of metastatic breast cancers. (A)** *In vitro* tube formation of human umbilical vein endothelial cells (HUVECs) after co-culture for indicated time with MDA-MB-231 cells either mocked transfected or transfected with indicated siRNAs or miRNA mimic (×100). **(B**-**D)** ELISA using the serum samples for comparison of VEGF-C levels in healthy volunteers, patients with benign lesions, and patients with breast cancers **(B)**, in patients with breast cancers in various stages **(C)**, and in patients with non-metastatic and metastatic breast cancers **(D)**.

### NFAT5 is a direct target of miR-568 in metastatic breast cancers

We next addressed the regulation of NFAT5 in metastatic breast cancers with particular interests in the responsible miRNAs, which abrogate gene expression at the post-transcriptional or translational level [17]. We searched for potential miRNAs which may target NFAT5, and identified miR-568 as a candidate regulator of NFAT5 (Figure 5A). Consistent with our previous findings in T lymphocytes [23], the expression of NFAT5 inversely correlated with miR-568 levels in breast cancer cell lines, with significantly lower miR-568 expression in highly invasive cell lines (Figure 5B). Suppression of miR-568 in MCF-7 cells caused the upregulation of NFAT5, whereas introduction of a miR-568 mimic dose-dependently decreased NFAT5 levels in MDA-MB-231 cells (Figure 5C). Consistently, miR-568 significantly inhibited the expression of a luciferase reporter gene fused to a specific wild-type but not mutated 3′ UTR of NFAT5, suggesting the direct targeting of NFAT5 by miR-568 (Figure 5D).

**Figure 5:** **miR-568 targets nuclear factors of activated T cells 5 (NFAT5) to regulate metastasis of breast cancers. (A)** Predicted binding sites of miR-568 on the 3′ UTR of NFAT5 mRNA. **(B)** qRT-PCR assay of breast cancer cell lines. Relative levels compared with GAPDH (for NFAT5) and U6 (for miR-568) were plotted. **(C)** Cells were transfected with miR-568 mimics, antagomiR-568, or scrambled control, followed by RT-PCR and western blot analysis. **(D)** Luciferase activity measured 24 h after co-transfection of HEK293 cells with miR-568 mimics and a pGL3 construct containing wild-type or mutant NFAT5 3′UTR regions encompassing the three predicted binding sites of miR-568. Data were normalized to cells co-transfected with scrambled miRNA and pGL3 vector. **(E)** qRT-PCR assays of MDA-MB-231 cells after transfection with indicated siRNAs. Relative levels compared with untransfected cells were plotted. **(F)** Transwell assays of cells transfected with the mimics or inhibitor of miR-568 or respective control. **(G)** Western blotting using the lysates of MDA-MB-231 cells transfected with control or miR-568 mimics. **(H)** H&E staining of primary tumors and the lung (left), and recorded incidence of lung metastases (right) by xenograft tumors derived from MDA-MB-231 cells modified with control (vector) or pre-miR-568-expressing recombinant lentiviruses. Arrows show the tumor boundary with black arrows indicating an invasive interface between the tumor and normal tissues. **(I)** qRT-PCR assay of clinically normal mammary tissues and breast cancer samples in Figure 1F. miR-568 levels normalized to U6 are plotted. All data are representative photographs or represent the mean ± SD of three replicates. *P <0.05.

The article "Nuclear factor of activated T cells 5 maintained by Hotair suppression of miR-568 upregulates S100 calcium binding protein A4 to promote breast cancer metastasis" was retracted in 2018. Reason: duplicated images.

The role of miR-568 in breast cancer metastasis was next evaluated. Similar to siRNA-mediated knockdown of NFAT5 or S100A4, miR-568 significantly decreased the levels of metastasis executioners (Figure 5E). Transfection with miR-568 significantly suppressed the invasiveness of MDA-MB-231 cells, while inhibition of miR-568 enhanced the invasion of MCF-7 cells in a transwell assay (Figure 5F). These results are consistent with the observation that introduction of miR-568 into MDA-MB-231 cells suppressed a mesenchymal phenotype and concurrently improved epithelial marker expression in these cells (Figure 5G). MDA-MB-231 cells were next infected with a control or pre-miR-568-expressing recombinant lentivirus, and were implanted subcutaneously in nude mice to allow for tumor development. Compared with the tumors derived from control cells, primary tumors that ectopically expressed miR-568 showed decreased invasion and infiltration of peripheral tissues (Figure 5H). Significantly lower frequency of lung metastasis was detected in xenograft tumor models with miR-568-overexpressing cells than in tumors from control breast cancer cells (Figure 5H). Clinically, miR-568 expression was much lower in metastatic breast cancers than in non-metastatic breast cancers cells or normal breast tissues (Figure 5I). These data suggest an essential role for miR-568 in suppressing distal metastasis probably by targeting NFAT5 in breast cancers.

The article "Nuclear factor of activated T cells 5 maintained by Hotair suppression of miR-568 upregulates S100 calcium binding protein A4 to promote breast cancer metastasis" was retracted in 2018. Reason: duplicated images.

### Hotair suppresses miR-568 to maintain NFAT5 expression in metastatic breast cancers

The lncRNA Hotair is an oncogenic RNA that is well known to be involved in the metastasis of various cancers [14]. We found that Hotair overexpression correlates with a high invasive capacity in breast cancer cell lines, while only modest expression of Hotair was detected in breast cancer cell lines with lower invasiveness (Figure 6A). Inhibition of Hotair by small interfering RNA (siRNA) dramatically impaired the invasiveness of breast cancer cells in a Matrigel assay (Figure 6B). The expression of Hotair was examined in clinical breast cancer samples (metastatic or non-metastatic) and paraneoplastic tissues. When grouped according to Hotair levels, patients with low Hotair expression showed significantly longer survival than those with high Hotair levels, suggesting that Hotair may be an independent prognostic factor of breast cancer (Figure 6C). These results are in agreement with the well-characterized pro-metastatic role of Hotair in cancer progression [14].

**Figure 6:** **Hotair epigenetically silences miR-568 in metastatic breast cancers. (A)** qRT-PCR assays of Hotair expression in breast cancer cell lines. Relative levels compared with MCF-10A cells were plotted. **(B)** qRT-PCR (left) and transwell (right) assays of MDA-MB-231 cells following transfection with the indicated siRNAs. Relative levels compared with mock-transfected cells were plotted. **(C)** Clinical breast cancer samples were divided into Hotair-low and -high groups (left), and the probablities of survival were plotted based on a review of in-patient records and a follow-up study (right). **(D)** Pearson correlation analysis of the relative expression levels of Hotair (normalized to glyceraldehyde-3-phosphate dehydrogenase, GAPDH) and miR-568 (normalized to U6) determined using qRT-PCR in 29 human breast cancer tissue samples. **(E)** qRT-PCR assay of MDA-MB-231 cells transfected with siRNAs targeting the indicated genes. **(F)** ChIPs were performed using the indicated antibodies, followed by amplification of the 5′ regulatory region of miR-568. All data are representative photographs or represent the mean ± SD of three replicates. *P <0.05, **P <0.01 compared with all other groups.

Hotair has been shown to negatively regulate a cohort of metastasis-suppressive genes via epigenetic modifications [13]-[15]. We next tested whether Hotair plays a regulatory role on miR-568 to potentiate metastasis in breast cancers. Indeed, a strong correlation between Hotair and miR-568 levels was observed in clinical breast cancers (Figure 6D). In addition, miR-568 was substantially elevated in response to knockdown of Hotair in metastatic breast cancer cells (Figure 6E). Given that Hotair recruits the PRC2 complex and LSD1, which are responsible for histone H3K27 methylation and H3K4 demethylation in target genomic loci, respectively [13], we silenced LSD1 and the PRC2 component EZH2 in breast cancer cells. Significant upregulation of miR-568 was observed in MDA-MB-231 cells in which either EZH2 or LSD1 was silenced, and inhibition of Hotair, EZH2, and LSD1 synergized to restore the expression of miR-568 (Figure 6E). The transcriptional start site (TSS) of the miR-568 gene was defined in the Ensembl database and the Eukaryotic Promoter Database (EPD) (Additional file 2: Figure S1A). This is consistent with a PolII promoter prediction 500 to 1000 bp upstream of the TSS by the UCSC Genome Browser (ENCODE), which also supports a high frequency of histone H3K27 methylation in this chromosomal region (Additional file 2: Figure S1B). Accordingly, we confirmed by ChIP the involvement of EZH2 and LSD1 binding, and consequently the histone H3K27 methylation and H3K4 demethylation in miR-568 suppression by Hotair in MDA-MB-231 cells (Figure 6F). Therefore, Hotair suppresses miR-568 via a previously established epigenetic mechanism involving recruitment of the PRC2 complex and histone H3K27 methylation in metastatic breast cancer.

The article "Nuclear factor of activated T cells 5 maintained by Hotair suppression of miR-568 upregulates S100 calcium binding protein A4 to promote breast cancer metastasis" was retracted in 2018. Reason: duplicated images.

## Discussion

Breast cancer metastasis is synergistically controlled by autonomous signaling within cancer cells and molecular signals originating from non-tumor cells within the changing microenvironment [4],[6]. In principle, cells in the primary tumor sense stringent conditions, such as nutrient deficiency, undergo intracellular signaling resulting in an altered gene expression profile, and initiate invasion and migration for ectopic survival [4],[5]. The canonical molecular machinery involved in the multi-step process of metastasis has been identified; however, it remains largely elusive how these metastasis executioners are regulated by intracellular signaling pathways controlled in response to a diverse set of stimuli [5],[6]. Here, we found that the transcriptional factor plays a key role in metastasis of breast cancers, potentiating EMT and migration of malignant cells by transcriptional activating of S100A4 and probably initiating angiogenesis of metastases via elevated secretion of VEGF-C. Non-coding RNAs are critically involved in the regulation of NFAT5 in that miR-568, which directly targets and suppresses NFAT5, was epigenetically silenced by the lncRNA Hotair.

The osmosensitive transcription factor NFAT5, also known as tonicity-responsive enhancer-binding protein (TonEBP), has been shown to participate in various physiological and pathological processes, particularly innate immunity and hypertension [24],[25]. In cancer progression, NFAT5 acts downstream of integrin signaling to promote invasiveness through unknown mechanisms [7],[20]. NFAT5 mediates integrin α6β4 signaling and induces the expression of the calcium-binding protein S100A4/metastasin to regulate breast cancer invasion [20],[26]. Consistent with these findings, we demonstrated that S100A4 and VEGF-C are direct targets of NFAT5 in highly invasive breast cancer cells. As a well-documented key player in metastasis, S100A4 is implicated in the regulation of a long list of genes acting at different stages of metastasis, based on its ability to interact with myosin, p53, and cytoskeletal proteins, as well as its ability to degrade extracellular matrix proteins [11]. In addition, VEGF-C enhances the permeability of vessels and induces angiogenesis and lymphangiogenesis, which expedite the local invasion, propogation, and colonization of neoplastic cells, making it a widely applicable indicator of pre-metastatic tumors [12]. While little is known about the mechanism through which S100A4 and VEGF-C may collaboratively promote metastasis, they exhibit coordinated expression in tumors, which is consistent with our findings that both are upregulated in metastatic breast cancers as target genes of NFAT5 [27].

The article "Nuclear factor of activated T cells 5 maintained by Hotair suppression of miR-568 upregulates S100 calcium binding protein A4 to promote breast cancer metastasis" was retracted in 2018. Reason: duplicated images.

Non-coding RNAs such as miRNAs and lnc RNAs have emerged as key mediators of signals underlying the malignant phenotype [14],[17]. Located on chromosome 3, the biological role of miR-568 has not been fully studied, which is in contrast to the numerous studies of miRNAs in carcinogenesis [17],[28]. The rare data available show that miR-568 correlates with the occurrence of diabetes. MiR-568 is also a circulating miRNA specifically produced by breast cancer cells [29],[30]. Conversely, we demonstrated here that intracellular miR-568 is downregulated in metastatic breast cancer cells by Hotair. It is possible that this discrepancy may result from differences in the ability of metastatic or localized breast tumors to secrete specific miRNAs, including miR-568, into extracellular compartments via exosomes or other vesicles. This putative mechanism, in addition to Hotair-triggered transcriptional repression, may further reduce cellular miR-568 in invasive breast cancer cells.

The lncRNA Hotair is well documented in promoting the metastasis of various malignancies and altering gene expression profiles by recruitment of PRC2 components and subsequent chromosomal gene silencing via coordinated histone H3K27 methylation and H3K4 demethylation [13]. Consistent with these reports, we found that Hotair impairs the expression of miR-568, a metastasis-suppressive miRNA, through the aforementioned epigenetic mechanism [13]. While there are so far very few miRNAs defined as targets of Hotair, our findings are in agreement with a previous report showing the localization of potential Hotair-responsive chromosomal regions by a genome-wide PRC2 occupancy analysis [14]. Although it is not known whether other metastasis-related miRNAs are suppressed by Hotair, or how Hotair is dramatically upregulated in metastatic breast cancer cells, our study suggests a novel pattern of metastatic cell signaling, in which Hotair represses a tumor suppressor miRNA and thereby maintains high levels of key transcription factors and their target gene products involved in metastasis.

The article "Nuclear factor of activated T cells 5 maintained by Hotair suppression of miR-568 upregulates S100 calcium binding protein A4 to promote breast cancer metastasis" was retracted in 2018. Reason: duplicated images.

The occurrence and progression of breast cancer is etiologically attributed to aberrant steroid hormone and human epidermal growth factor receptor (HER) signaling, and breast cancers are thereby clinically classified by the expression of estrogen receptors (ER), progesterone receptors (PR), and HER2 [31]-[33]. Whereas therapeutics targeting these markers have been developed and have benefited a large population of patients, triple-negative breast cancers usually represent a more aggressive pathological type with a poor prognosis, suggesting the critical involvement of pro-survival and pro-metastasis signaling pathways other than ER/PR and HER2 pathways [34]-[36]. In this regard, whether Hotair accumulation results from aberrant upstream signaling is unknown, nor is whether and how miR-568 or NFAT5 may be controlled by alternative signaling, for example, the well-defined pathways involved in mammary malignancy [14]. The high expression of lncRNA Hotair is independent of known clinical risk factors, for example, tumor stage and HER2 or hormone receptor status [14]. As a evolutionarily conserved lncRNA, which is also involved in maintenance of chromatin structure in normal cells, Hotair might become abundant in stochastic clones that consequently gain survival and migration advantages over other cells and potentiate distal metastasis, as proposed previously for the well-documented cancer-initiating cells [36]. Although this hypothesis is consistent with the observation that Hotair signaling promotes EMT, a characteristic of cancer stem cells, further evidence is needed to confirm that Hotair is a driver of *de novo* carcinogenesis and is indispensable for the development of metastatic loci [36],[37].

## Conclusion

NFAT5 promotes breast cancer progression by transcriptionally activating S100A4 and VEGF-C, whereas the redundant NFAT5 is maintained by Hotair-elicited epigenetic silencing of miR-568. Our finding that Hotair signals through miRNA(s) and key transcriptional factor(s) to affect the expression of metastatic genes provides novel insights into molecular mechanisms of metastasis involving non-coding RNAs, and thus has implications for the development of novel therapeutic approaches targeting metastatic breast cancers.

The article "Nuclear factor of activated T cells 5 maintained by Hotair suppression of miR-568 upregulates S100 calcium binding protein A4 to promote breast cancer metastasis" was retracted in 2018. Reason: duplicated images.

## Author contributions

JTL and YLZ designed and performed most *in vitro* experiments. LFW and TY collected clinical samples and conducted investigations on these samples. WL and LW generated DNA constructs including the luciferase reporter plasmids. YLM technically optimized the studies on gene expression and cell behavior. NNL and XSZ helped analyze the clinical data. JZ, FY and CFG substantially provided essential suggestions on the proposal and helped draft the work. LTJ and AGY analyzed the data and wrote the paper. All authors read and approved the final manuscript.

## Additional files

## Electronic supplementary material

Additional file 1: Table S1.: Primers used for PCR amplification and targeting sites of siRNAs. (DOC 47 KB)

Additional file 2: Figure S1.: The genomic context and histone modifications of human miR-568 transcript. **(A)** Schematic presentation indicating the transcript of the miR-568 gene in the eukaryotic promoter database (EPD). **(B)** ENCODE annotation of the miR-568 gene in various cell lines showing characterized histone modifications including H3K27 trimethylation upstream of the transcriptional start site. (PDF 373 KB)

Below are the links to the authors’ original submitted files for images.

Authors’ original file for figure 1

Authors’ original file for figure 2

Authors’ original file for figure 3

Authors’ original file for figure 4

Authors’ original file for figure 5

Authors’ original file for figure 6

## Abbreviations

bp: base pairs
ChIP: chromatin immunoprecipitation
DAPI: 4′,6-diamidino-2-phenylindole
DMEM: Dulbecco’s modified Eagle’s medium
ELISA: enzyme-linked immunosorbent assay
EMT: epithelial-mesenchymal transition
FBS: fetal bovine serum
GAPDH: glyceraldehyde-3-phosphate dehydrogenase
H&E: hematoxylin and eosin
HER: human epidermal growth factor receptor
HUVEC: human umbilical vein endothelial cell
LncRNA: long non-coding RNA
miRNA: microRNA
MMP: matrix metalloproteinase
NFAT5: nuclear factors of activated T cells 5
PRC2: polycomb repressive complex 2
shRNA: short hairpin RNA
siRNA: short interfering RNA
SP: strepavidin-peroxidase
TSS: transcriptional start site
UTR: untranslated region
VEGF-C: vascular endothelial growth factor C
